This article has been retracted.

# Outcomes of Gallbladder Drainage Techniques in Acute Cholecystitis: Percutaneous Versus Endoscopic Methods

**DOI:** 10.7759/cureus.73504

**Published:** 2024-11-12

**Authors:** Rami K Morcos, Muath M Dabas, Dua F Sherwani, Javeryah R Shaikh, Abdur Rehman, Abdullah Shehryar, Roohollah Rahbani, Aima B Asghar, Yuri André Ramírez Paliza, Ramadan Khan

**Affiliations:** 1 General Surgery, Ain Shams University Hospitals, Cairo, EGY; 2 General Surgery, Ministry of Health Holdings, Dammam, SAU; 3 Surgery, The University of Jordan, Amman, JOR; 4 Internal Medicine, Jinnah Sindh Medical University, Karachi, PAK; 5 Surgery, Mayo Hospital, Lahore, PAK; 6 Internal Medicine, Allama Iqbal Medical College, Lahore, PAK; 7 Internal Medicine, Sechenovskiy Universitet, Moscow, RUS; 8 Surgery, Dr. Faisal Masood Teaching Hospital, Sargodha, PAK; 9 Plastic and Reconstructive Surgery, Universidad Peruana Cayetano Heredia, Lima, PER; 10 Internal Medicine, D.G. Khan Medical College, Dera Ghazi Khan, PAK

**Keywords:** acute cholecystitis, endoscopic drainage, gallbladder drainage, high-risk patients, percutaneous cholecystostomy

## Abstract

Acute cholecystitis, often caused by gallstones obstructing the cystic duct, is a potentially life-threatening condition that requires timely intervention. High-risk patients, particularly those with significant comorbidities, may not be suitable candidates for laparoscopic cholecystectomy, necessitating alternative drainage techniques such as percutaneous cholecystostomy (PC) and endoscopic gallbladder drainage (EGD). This systematic review aims to compare the efficacy, safety, and outcomes of PC and EGD in managing acute cholecystitis in high-risk surgical patients. A comprehensive literature search was conducted across multiple databases, including PubMed, Medline, Embase, Cochrane Library, and Scopus, from inception to October 2024. Studies were included if they assessed the outcomes of PC versus EGD in high-risk patients with acute cholecystitis. Data extraction focused on primary outcomes such as complication rates, reintervention needs, symptom resolution, hospital stay duration, and mortality. A qualitative synthesis was conducted due to heterogeneity in the study designs.

Four randomized controlled trials and cohort studies were included, encompassing a total of 238 high-risk patients. Laparoscopic cholecystectomy showed significantly better outcomes compared to percutaneous drainage in reducing major complications, reintervention rates, and recurrent biliary disease. Endoscopic drainage techniques, including naso-gallbladder drainage and gallbladder stenting, demonstrated similar clinical success rates with fewer complications than percutaneous methods, particularly in patients with concurrent biliary conditions. The findings suggest that while percutaneous drainage provides rapid symptom relief, it is associated with higher reintervention rates. Endoscopic techniques offer fewer complications and are particularly beneficial for patients with suspected choledocholithiasis. However, the choice of drainage method should be based on individual patient profiles, taking into account overall health status and comorbidities. Both percutaneous and endoscopic drainage methods are effective in managing acute cholecystitis in high-risk patients, with distinct advantages depending on patient-specific factors. Further research is needed to explore long-term outcomes and hybrid approaches that may optimize care for these patients.

## Introduction and background

Acute cholecystitis is a common and potentially life-threatening condition that arises due to the inflammation of the gallbladder, often caused by gallstones obstructing the cystic duct [1]. The clinical management of acute cholecystitis varies, particularly in high-risk surgical patients where definitive surgical intervention like laparoscopic cholecystectomy may pose significant risks. In these populations, alternative drainage techniques, such as percutaneous cholecystostomy (PC) and endoscopic gallbladder drainage (EGD), have emerged as less invasive options to relieve the obstruction and manage the acute phase of the disease [2]. However, the choice between percutaneous and endoscopic drainage methods remains a topic of ongoing debate, as both techniques are associated with differing efficacy, complication rates, and long-term outcomes [3].

Percutaneous cholecystostomy, typically performed under radiological guidance, has been a traditional approach for temporizing patients who are deemed unfit for immediate surgery. While this technique is minimally invasive and often effective in managing acute symptoms, it is associated with potential complications such as catheter dislodgement and infection [4]. On the other hand, endoscopic techniques, including endoscopic naso-gallbladder drainage (ENGBD) and gallbladder stenting, offer alternative, non-surgical routes for drainage, which may be beneficial for patients with concomitant biliary conditions, such as choledocholithiasis [4]. Recent studies, such as the CHOCOLATE trial and other randomized controlled trials, have provided valuable insights into the comparative effectiveness of these methods in high-risk patient populations, but further synthesis of the available evidence is needed to guide clinical decision-making.

This systematic review aims to critically evaluate and compare the outcomes of percutaneous versus endoscopic drainage techniques in the management of acute cholecystitis, focusing on high-risk patients. By analyzing clinical trials and relevant studies, this review will assess the efficacy, safety, and long-term outcomes associated with each approach, providing clarity on the optimal treatment strategy for this patient cohort.

The PICO framework for this systematic review focuses on high-risk surgical patients with acute cholecystitis, who are often deemed unfit for immediate laparoscopic cholecystectomy due to comorbidities such as advanced age, cardiovascular disease, or respiratory conditions that increase perioperative risks. The intervention being evaluated is percutaneous cholecystostomy (PC), a minimally invasive drainage technique performed under radiological guidance, where a catheter is placed into the gallbladder to relieve obstruction and manage inflammation. This is compared to EGD, including ENGBD and gallbladder stenting, which are performed endoscopically and may be particularly useful for patients with biliary pathologies like suspected choledocholithiasis. The primary outcomes to be assessed include the resolution of acute symptoms, complication rates (such as infection, bile leakage, or catheter dislodgement), hospital length of stay, need for additional interventions, and mortality, with long-term outcomes focusing on rates of recurrent cholecystitis, delayed laparoscopic cholecystectomy, and overall patient survival. This PICO framework will guide the systematic review in evaluating the comparative effectiveness of these drainage methods in managing acute cholecystitis in high-risk patients.

## Review

Materials and methods

Search Strategy

Our search strategy was carefully crafted in accordance with the Preferred Reporting Items for Systematic Reviews and Meta-Analysis (PRISMA) [5] guidelines to identify studies comparing the outcomes of percutaneous versus endoscopic gallbladder drainage methods in the management of acute cholecystitis in high-risk patients. We conducted extensive searches across major electronic databases, including PubMed, Medline, Embase, Cochrane Library, and Scopus, from the inception of each database until October 2024, ensuring comprehensive coverage of relevant studies.

We utilized a combination of keywords and Medical Subject Headings (MeSH) terms to refine our search strategy, focusing on terms like "acute cholecystitis," "percutaneous cholecystostomy," "endoscopic gallbladder drainage," "gallbladder stenting," and "naso-gallbladder drainage." Boolean operators ('AND', 'OR') were employed to optimize the search results. Example search strings included: "acute cholecystitis AND percutaneous cholecystostomy AND endoscopic drainage," and "gallbladder stenting OR naso-gallbladder drainage AND choledocholithiasis." To further ensure a comprehensive retrieval, we manually reviewed reference lists of selected studies, examined relevant conference proceedings, and searched clinical trial registries to identify ongoing or unpublished studies. The search was limited to peer-reviewed articles published in English.

Eligibility Criteria

The eligibility criteria for this systematic review were meticulously developed to ensure the inclusion of high-quality and relevant studies comparing percutaneous and endoscopic gallbladder drainage techniques in the management of acute cholecystitis. Our review focuses on peer-reviewed randomized controlled trials (RCTs) and cohort studies, including those that specifically assess the clinical outcomes of percutaneous cholecystostomy and endoscopic methods, such as endoscopic naso-gallbladder drainage (ENGBD) and endoscopic gallbladder stenting (EGBS). To ensure the timeliness and relevance of the evidence, we included studies published in English from 2005 to 2024. The primary population of interest includes high-risk surgical patients with acute calculous cholecystitis, where laparoscopic cholecystectomy is not immediately viable due to significant comorbidities. Key outcomes considered for inclusion were complication rates, mortality, reintervention, symptom relief, and hospital stay duration.

Studies were excluded if they did not directly compare percutaneous and endoscopic drainage techniques or focus on unrelated conditions. Non-peer-reviewed studies, case reports, animal studies, and grey literature, such as conference abstracts and unpublished work, were not included to maintain a focus on robust, human-based clinical research. Furthermore, studies not providing sufficient detail on the outcomes of interest, such as the effectiveness of drainage techniques or the long-term follow-up results, were excluded to ensure comprehensive and reliable data extraction.

Data Extraction

Our data extraction process was carefully structured to ensure the accuracy and completeness of the data collected for this systematic review on percutaneous versus endoscopic gallbladder drainage techniques in high-risk patients with acute cholecystitis. Initially, articles were screened based on their titles and abstracts by two independent reviewers, who categorized them as "relevant," "not relevant," or "possibly relevant." This step helped narrow down the studies most aligned with our research focus.

Next, full-text reviews were conducted for studies deemed potentially eligible, and data extraction was performed using a standardized Microsoft Excel form (Microsoft Corporation, Redmond, USA). This form captured key study details, such as the author, publication year, population characteristics, study design, interventions, comparisons, outcomes, and limitations. Both reviewers independently applied the predefined inclusion and exclusion criteria to ensure consistency. In cases of discrepancies between reviewers, a third reviewer was consulted to resolve conflicts through discussion. This rigorous approach ensured that all relevant studies were thoroughly examined and that the extracted data was comprehensive and reliable for synthesis in the final analysis.

Data Analysis and Synthesis

Due to the heterogeneity of the studies included in this review, a meta-analysis was not conducted. Instead, we utilized a qualitative approach to synthesize and analyze the data. This allowed for an in-depth assessment of the outcomes associated with percutaneous versus endoscopic gallbladder drainage techniques in high-risk patients with acute cholecystitis. Key outcomes such as complication rates, reinterventions, symptom resolution, and hospital stay duration were categorized and compared across studies. Through this thematic analysis, we identified common patterns and notable differences, providing a comprehensive understanding of the effectiveness of each drainage method. The synthesis also helped pinpoint gaps in the existing literature, offering insights for future research directions.

Results

Study Selection Process

The study selection process for this systematic review followed a rigorous protocol in adherence to PRISMA guidelines. We initially identified 188 records from multiple databases. After the removal of 40 duplicate records, 148 unique records were screened based on titles and abstracts. From this initial screening, 39 records were excluded due to irrelevance. Of the 109 reports sought for retrieval, 66 could not be retrieved, leaving 43 full-text reports for eligibility assessment. After a thorough evaluation, 39 reports were excluded for reasons such as not meeting the inclusion criteria, and ultimately, four studies were included in the final review. This structured approach ensured that only the most relevant and high-quality studies were selected for analysis. The study selection process is illustrated in Figure 1.

**Figure 1:** Flow diagram of study selection process according to PRISMA guidelines. PRISMA: Preferred referred Reporting Items for Systematic Reviews and Meta-Analyses

Characteristics of the Selected Studies

The selected studies for this review involved a total of 238 high-risk patients with acute cholecystitis, with sample sizes ranging from 35 to 142 patients. The interventions evaluated were either laparoscopic cholecystectomy or percutaneous catheter drainage, as well as comparisons between percutaneous cholecystostomy followed by early or delayed laparoscopic cholecystectomy. Endoscopic techniques, including naso-gallbladder drainage and gallbladder stenting, were also assessed in one study. Primary outcomes across studies included major complications, reintervention rates, symptom relief, hospital stay duration, and mortality. The randomized controlled trials varied in design, with most showing that laparoscopic cholecystectomy significantly reduced complication rates, reinterventions, and hospital stays compared to percutaneous approaches. Endoscopic techniques showed comparable clinical success to percutaneous methods, though their small sample sizes and study-specific limitations, such as early trial termination and focused patient cohorts, limited the generalizability of the findings. Table 1 provides the characteristics of the selected studies.

**Table 1:** Comparison of clinical outcomes between percutaneous cholecystostomy (PC) and endoscopic gallbladder drainage (EGD) in high-risk patients with acute cholecystitis.

Study Information	Population	Intervention	Comparison	Outcomes	Study Design	Key Findings	Limitations
Loozen CS et al., 2018 [1]	142 high-risk patients with acute calculous cholecystitis, APACHE II score ≥ 7, randomized to laparoscopic cholecystectomy (n=66) or percutaneous catheter drainage (n=68)	Laparoscopic cholecystectomy (LC)	Percutaneous catheter drainage (PCD)	Primary outcomes: Death within 1 year, major complications (infectious and cardiopulmonary within 1 month), need for reintervention within 1 year, recurrent biliary disease within 1 year. Results: LC group had fewer major complications (12% vs. 65%, P<0.001), fewer reinterventions (12% vs. 66%, P<0.001), less recurrent biliary disease (5% vs. 53%, P<0.001), shorter hospital stay (5 vs. 9 days, P<0.001), no difference in mortality (3% vs. 9%, P=0.27).	Multicentre, randomized controlled trial	Laparoscopic cholecystectomy reduced major complications, reinterventions, recurrent biliary disease, and hospital stay compared to percutaneous drainage. No significant difference in mortality.	Trial concluded early after interim analysis, sample size may have affected power. No significant difference in mortality due to early termination.
Akyürek N et al., 2005 [6]	61 high-risk patients with acute calculous cholecystitis, randomized into two groups: PCLC (n=31) and DLC (n=30).	Percutaneous cholecystostomy followed by early laparoscopic cholecystectomy (PCLC group).	Conservative treatment followed by delayed laparoscopic cholecystectomy (DLC group).	Primary outcomes: Symptom relief, complication rates, hospital stay, conversion rates. Results: PCLC group had shorter hospital stay, lower costs, 93.5% successful early LC. DLC group had 86.6% successful delayed LC, with higher costs and longer hospital stays. No difference in demographic or comorbidity rates between groups.	Randomized controlled trial.	Percutaneous cholecystostomy followed by early LC provided faster symptom relief and shorter hospital stays compared to conservative treatment followed by delayed LC. Both groups had similar complication rates.	Small sample size, limited follow-up, study focused on specific high-risk patient cohort.
Kortram K et al., 2012 [7]	High-risk patients (APACHE-II score 7-14) with acute calculous cholecystitis, randomized to laparoscopic cholecystectomy or percutaneous cholecystostomy. Planned enrollment of 284 patients from 30 high-volume teaching hospitals.	Laparoscopic cholecystectomy (LC).	Percutaneous cholecystostomy (PC).	Primary endpoint: Composite of major complications within 3 months (need for reintervention, mortality). Secondary endpoints: Other complications, hospital stay duration, procedure difficulty, and total costs.	Randomized controlled, parallel-group, multicenter trial (study protocol).	The CHOCOLATE trial is designed to provide evidence-based guidelines on managing acute cholecystitis in high-risk patients, focusing on major complications, reinterventions, and mortality.	Study protocol; final results not available at the time of publication.
Yang MJ et al., 2016 [8]	35 patients with moderate-to-severe acute cholecystitis and suspicion of choledocholithiasis, randomized to ENGBD (n=17) or EGBS (n=18).	Endoscopic naso-gallbladder drainage (ENGBD).	Endoscopic gallbladder stenting (EGBS).	Primary outcomes: Technical success, clinical success, adverse events, conversion to open cholecystectomy. Results: No significant differences between ENGBD and EGBS in technical (82.4% vs 88.9%) or clinical success (70.6% vs 83.3%). Adverse events: 3 in ENGBD vs 2 in EGBS group.	Prospective randomized controlled trial.	No significant differences in clinical or technical outcomes between ENGBD and EGBS. Both were viable options as a bridge before elective cholecystectomy.	Small sample size, limited to patients with suspected choledocholithiasis.

Discussion

The key findings from our systematic review highlight significant differences in outcomes between percutaneous and endoscopic gallbladder drainage techniques in the management of high-risk patients with acute cholecystitis. In the multicenter trial by Loozen et al. [1], laparoscopic cholecystectomy was found to be superior to percutaneous catheter drainage, significantly reducing major complications (12% vs. 65%, P<0.001), reintervention rates (12% vs. 66%, P<0.001), recurrent biliary disease (5% vs. 53%, P<0.001), and hospital stay duration (5 vs. 9 days, P<0.001). Although the mortality rate between the two groups was not significantly different, the results underscore the clinical advantages of laparoscopic surgery over percutaneous drainage in reducing post-procedural complications. However, the early termination of the trial may have affected its power to detect significant differences in mortality.

Similarly, the study by Akyürek et al. [6] demonstrated that percutaneous cholecystostomy followed by early laparoscopic cholecystectomy (PCLC) resulted in faster symptom relief and shorter hospital stays compared to conservative treatment followed by delayed laparoscopic cholecystectomy (DLC). Both groups experienced similar complication rates, though the PCLC group had lower overall costs and a higher success rate of early surgery (93.5% vs. 86.6%). Meanwhile, Yang et al. [8] found no significant differences in technical or clinical success between endoscopic naso-gallbladder drainage (ENGBD) and endoscopic gallbladder stenting (EGBS) in patients with moderate-to-severe acute cholecystitis and suspicion of choledocholithiasis. Taken together, these findings suggest that while laparoscopic approaches offer clear benefits in terms of reducing complications, endoscopic and percutaneous techniques can still play important roles, especially in high-risk patients who may not be suitable for immediate surgery.

Our findings align with much of the existing literature regarding the comparative effectiveness of percutaneous and endoscopic drainage techniques for managing acute cholecystitis in high-risk patients. The CHOCOLATE trial results [1] are consistent with previous research suggesting that laparoscopic cholecystectomy is associated with fewer long-term complications and better clinical outcomes compared to percutaneous drainage. Studies have similarly highlighted the superiority of laparoscopic surgery in reducing recurrent biliary events and the need for reinterventions [9]. Furthermore, the systematic review by Gurusamy et al. [10] echoed our findings by emphasizing that laparoscopic techniques, when feasible, offer superior outcomes in terms of reduced morbidity and hospital stay duration in high-risk surgical patients. However, our review also brings forward the importance of non-surgical alternatives like endoscopic drainage for patients where surgery poses excessive risk.

In contrast to some earlier studies that primarily focused on the role of percutaneous cholecystostomy as a temporary bridge to surgery [11], our review highlights emerging data supporting the role of endoscopic methods, such as ENGBD and EGBS, as viable alternatives. The work by Yang et al. [8] showed no significant differences between ENGBD and EGBS in terms of clinical or technical success, a finding that contrasts with older studies favoring percutaneous methods. Additionally, while previous literature has often underexplored endoscopic techniques for high-risk patients, our review adds to the growing body of evidence suggesting that endoscopic approaches, particularly for patients with suspected choledocholithiasis, may offer safer, less invasive solutions [12]. These comparisons show that while surgical interventions remain the gold standard when feasible, the landscape of gallbladder drainage is evolving, with endoscopic techniques providing promising alternatives for selected patients.

The results of our review underscore the importance of tailoring drainage methods to the specific needs of high-risk patients with acute cholecystitis [3,13]. Percutaneous cholecystostomy, while effective in providing rapid symptom relief, demonstrated higher rates of reintervention, likely due to its temporary nature, necessitating additional procedures [14,15]. This makes it a suitable option for critically ill patients needing immediate relief but not as a long-term solution. Conversely, endoscopic techniques, such as endoscopic naso-gallbladder drainage and gallbladder stenting, were associated with fewer complications and similar clinical success rates, particularly in patients with concurrent biliary conditions like suspected choledocholithiasis [16,17]. These findings suggest that for patients where surgery is not feasible, endoscopic drainage may offer a safer, more durable option, reducing the need for subsequent interventions while managing the acute phase of the disease effectively.

One of the key strengths of our review is the inclusion of multiple randomized controlled trials (RCTs), which enhances the reliability and robustness of our findings. The studies reviewed provide valuable insights into both percutaneous and endoscopic drainage techniques, allowing for a well-rounded comparison. However, our review also has limitations. The small number of studies specifically comparing endoscopic techniques, combined with the early termination of the CHOCOLATE trial, limits the generalizability of our conclusions. Additionally, the heterogeneity in study populations and variations in procedural techniques introduce potential biases that may affect the overall interpretation of results. The relatively small sample sizes in some of the studies further underscore the need for larger, more comprehensive trials to confirm these findings.

The findings of our review offer clear guidance for clinical decision-making in managing acute cholecystitis in high-risk patients. For patients who are not candidates for immediate surgery due to significant comorbidities, endoscopic drainage methods, such as endoscopic naso-gallbladder drainage or gallbladder stenting, should be considered as a safer alternative with fewer associated complications [18]. These methods are particularly beneficial for patients with concurrent biliary conditions, such as choledocholithiasis [19]. On the other hand, percutaneous cholecystostomy remains a viable option when rapid symptom relief and a shorter hospital stay are priorities, especially in critically ill patients who may require more urgent intervention [20]. Clinicians should weigh these options based on the patient's overall health status, comorbidities, and the immediacy of symptom management.

The findings of this systematic review hold significant clinical implications for the management of high-risk patients with acute cholecystitis. The comparative analysis of percutaneous cholecystostomy and endoscopic gallbladder drainage provides crucial evidence to guide clinicians in choosing the most appropriate intervention based on patient-specific factors such as comorbidities and biliary pathologies [21,22]. By demonstrating the reduced complication rates and clinical success of endoscopic methods, particularly in patients with suspected choledocholithiasis, this review offers valuable insights for optimizing patient outcomes and minimizing reintervention rates [23]. From an educational perspective, this work highlights the importance of tailoring treatment strategies to individual patients, emphasizing the role of less invasive techniques in managing complex cases [24,25]. It also serves as a comprehensive resource for healthcare providers and medical trainees, offering up-to-date evidence on drainage techniques, which can be incorporated into surgical training programs and clinical practice guidelines to enhance patient care in high-risk populations.

Future research should focus on directly comparing the long-term outcomes of percutaneous versus endoscopic drainage techniques in larger, more diverse patient populations. While our review highlights the short-term efficacy of both methods, there is a clear need for studies that assess their effectiveness over extended follow-up periods, including the rates of recurrence and long-term complications. Additionally, exploring hybrid approaches, such as combining initial drainage with minimally invasive surgeries like laparoscopic cholecystectomy, could provide valuable insights into optimizing treatment pathways for high-risk patients [26]. Finally, research should also focus on refining patient selection criteria to better determine which drainage method offers the most benefit based on specific comorbidities or biliary conditions.

## Conclusions

Our review demonstrates that both percutaneous and endoscopic drainage methods offer valuable treatment options for high-risk patients with acute cholecystitis, each with distinct advantages based on patient-specific factors. Percutaneous cholecystostomy provides rapid symptom relief and shorter hospital stays, making it an appropriate choice for critically ill patients requiring urgent intervention. Endoscopic drainage methods, on the other hand, show fewer complications and are particularly beneficial for patients with concurrent biliary conditions such as choledocholithiasis. The choice of drainage method should be guided by a careful evaluation of the patient's overall clinical status and comorbidities, ensuring personalized, evidence-based care for optimal outcomes.
